The article "Whether Economic Freedom Is Significantly Related to Death of COVID-19" was published in 2020. Journal: J Healthc Eng.

# Whether Economic Freedom Is Significantly Related to Death of COVID-19

**DOI:** 10.1155/2020/6660160

**Published:** 2020-12-09

**Authors:** Ray-Ming Chen

**Affiliations:** School of Mathematics and Statistics, Baise University, 21 Zhongshan No. 2 Road, Baise, Guangxi, China

## Abstract

COVID-19 has caused a huge mayhem globally. Different economic freedom leads to different performances of a country's reaction to the pandemic. We study 164 countries and apply mathematical and statistical approaches to tackle the problem: whether economic freedom has a significant impact on the death of COVID-19. We devise a metric, some norms, and some orderings to construct an absolute reference and the actual relation via binary sequences. Then, we use the theoretical binary sequences to construct a probability distribution which linearises the strength of relation between economic freedom and death of COVID-19. Then, the actual relation from the data analysis provides an evidence to the hypothetical testing. Our analysis and model show that there is no significant relation between economic freedom and death of COVID-19.

## 1. Introduction

Due to COVID-19 pandemic, there are many fatalities across the world. Many countries are baffled by whether to open the market or impose lockdown [1–3]. It creates a huge chaos in either economic or social stability [4, 5]. This motivates us to study the relation between economic freedom and the death rate or tolls of COVID-19. We locate 164 countries from some datasets [6, 7]—because some of the countries lack statistics of either the economic freedom or the death information regarding COVID-19. Then, we use a series of mathematical and statistical approaches to reach a conclusion. For the mathematical part, we define a new concept of metric *d* which could measure the difference between the scoring structures—this is hardly the case if one adopts the usual Euclidean metric. For reference purpose, one fixes the referential structure $\overset{⟶}{e}$ (or scoring system) first. Then, one could compute the distances between all the (sampled) multivalued data *N* points $\left\{{\overset{⟶}{v}}_{i}:1\leq i\leq N\right\}$ and *I*, i.e., $\left\{d\left(\overset{⟶}{e},{\overset{⟶}{v}}_{i}\right):1\leq i\leq N\right\}$. Based on these distances, we could then create an ordering for $\left\{{\overset{⟶}{v}}_{i}:1\leq i\leq N\right\}$ with respect to the referential structure $\overset{⟶}{e}$.

## 2. Modelling

### 2.1. Notations and Symbols

For a vector $\overset{⟶}{w}$, we use $\left|\overset{⟶}{w}\right|$ to denote its length; for any set *H*, we use |*H*| to denote its size (cardinality). Moreover, we use $\overset{⟶}{w}\left(j\right)$ to denote the *j*-th element in $\overset{⟶}{w}$. Let $\overset{⟶}{b}$ denote a binary vector, i.e., each element in $\overset{⟶}{b}$ is either 0 or 1. Let *𝔹*_*k*_ denote the set of all the binary vectors with total length *k*. Let *ℂ*={*C*_1_, *C*_2_,…, *C*_*m*_} be a set of countries. Let *A*_*ef*_={*A*_1_, *A*_2_,…, *A*_*n*_} be a set of attributes of economic freedom (regarded as independent variables). Let *B*_*j*_ be a set of result (regarded as dependent variables). Each time we fix one *B*_*j*_ to study the relation between the attributes and *B*_*j*_. In this article, we restrict our attribute values to be numerical numbers. The theoretical table is shown in Table 1, and for the actual forms, one could refer to Sections 3.2.1 and 3.2.2.

We use the notations $\overset{⟶}{C_{i}}=\left(a_{i1},a_{i2},\ldots ,a_{im}\right)$; $\overset{⟶}{A_{i}}=\left(a_{1i},a_{2i},\ldots ,a_{mi}\right)$; and $\overset{⟶}{B_{i}}=\left(b_{1i},b_{2i},\ldots ,b_{mi}\right)$.

### 2.2. Binary Subvectors and Norm

**Definition 1 .**

(subvectors). Suppose $\overset{⟶}{b}$ is a binary vector. We use $\text{Sub}\left(\overset{⟶}{b}\right)$ to denote all its truncated subvectors consisting of only 1.

**Example 1 .**

Suppose $\overset{⟶}{b}=\left(1,0,1,0,0,1,1,1,0,1,1,0,1,0,1,1,0,0,0,1,1,0,1,0\right)$. Then, $\text{Sub}\left(\overset{⟶}{b}\right)=\left\{\left(1\right),\left(1\right),\left(1,1,1\right),\left(1,1\right),\left(1\right),\left(1,1\right),\left(1,1\right),\left(1\right)\right\}$.

We simply abbreviate it as $\text{Sub}\left(\overset{⟶}{b}\right)=1^{1}1^{1}1^{3}1^{2}1^{1}1^{2}1^{2}1^{1}$. Indeed $\text{Sub}\left(\overset{⟶}{b}\right)$ reveals the structure of an independent-dependent variable relation.

**Definition 2 .**

(binary norm). For any binary vector $\overset{⟶}{b}=\left(b_{1},b_{2},\ldots ,b_{k}\right)$ with $\text{Sub}\left(\overset{⟶}{b}\right)=1^{n_{1}}1^{n_{2}},\ldots ,1^{n_{t}}$, define a binary norm $\left\|\overset{⟶}{b}\right\|=\left(2^{0}+2^{1}+\cdots +2^{n_{1}-1}\right)+\left(2^{0}+2^{1}+\ldots +2^{n_{2}-1}\right)+\cdots +\left(2^{0}+2^{1}+\cdots +2^{n_{t}-1}\right)$.

One could, according to real situations, adopt other numbers (for example, replace 2 with other numbers) or other forms other than the one provided here.

**Claim 1 .**

$\left\|\overset{⟶}{b}\right\|=\left(2^{n_{1}}+2^{n_{2}}+\cdots +2^{n_{t}}\right)-t$.

**Proof**

It follows immediately from the definition.

**Definition 3 .**

(linear ordering on *𝔹*_*k*_). ${\overset{⟶}{b}}_{1}\geq {\overset{⟶}{b}}_{2}$ if and only if $\left\|{\overset{⟶}{b}}_{1}\right\|\geq \left\|{\overset{⟶}{b}}_{2}\right\|$, for all ${\overset{⟶}{b}}_{1},{\overset{⟶}{b}}_{2}\in {𝔹}_{k}$.

**Example 2 .**

If ${\overset{⟶}{b}}_{1}=\left(1,0,1,1,1,0,0,1,1,0,1,0,1\right),{\overset{⟶}{b}}_{2}=\left(1,0,0,0,0,1,1,0,0,1,1,1,1\right)$, then $\left\|{\overset{⟶}{b}}_{1}\right\|=\left(2^{0}\cdot 1\right)+\left(2^{0}\cdot 1+2^{1}\cdot 1+2^{2}\cdot 1\right)+\left(2^{0}\cdot 1+2^{1}\cdot 1\right)+\left(2^{0}\cdot 1\right)+\left(2^{0}\cdot 1\right)=13$ and $\left\|{\overset{⟶}{b}}_{2}\right\|=\left(2^{0}\cdot 1\right)+\left(2^{0}\cdot 1+2^{1}\cdot 1\right)+\left(2^{0}\cdot 1+2^{1}\cdot 1+2^{2}\cdot 1+2^{3}\cdot 1\right)=19$. Thus, ${\overset{⟶}{b}}_{2}\leq {\overset{⟶}{b}}_{1}$.

**Remark 1 .**

A binary norm indeed serves an important technique in revealing the relation between dependent and independent variables. Given two pairs (*x*_1_, *y*_1_) and (*x*_2_, *y*_2_) of numerical data with *x*_1_ ≠ *x*_2_, if (*x*_2_ − *x*_1_) · (*y*_2_ − *y*_1_) > 0 (i.e., they act proportionally), we associate it with a value 1 to indicate such relation and 0, otherwise (i.e., they act inversely). Such mechanism gives a way to look into the fundamental relation between *X* and *Y* variables. This kind of analysis is in particular useful when the precision of the data is questionable or when the actual numbers are unknown or more suitable to be interpreted via ranks.

**Example 3 .**

(sign vector). Suppose *D*=((2,4), (3,2), (5,8), (7,9), (4,2), (3,8)), a set of ordered vectors. Then, we could associate *D* with a sign vector $\overset{⟶}{v}=\left(0,1,1,1,0\right)$ via Remark 1.

**Definition 4 .**

(relational vector). Suppose that $\overset{⟶}{b}$ is a sign vector; we associate it with a relational vector $\text{Rel}\left(\overset{⟶}{b}\right)$ whose *i*-th element is assigned 1 iff $\overset{⟶}{b}\left(i\right)=\overset{⟶}{b}\left(i+1\right)$ and 0, otherwise.

**Example 4 .**

Let us continue with Example 3. We could compute its relational vector $\text{Rel}\left(\overset{⟶}{v}\right)=\left(0,1,1,0\right)$, and thus $\text{Sub}\left(\text{Rel}\left(\overset{⟶}{v}\right)\right)=1^{2}$ and $\left\|\text{Sub}\left(\text{Rel}\left(\overset{⟶}{v}\right)\right)\right\|=3$. The higher the value of the norm is, the closer the relation between the dependent and independent variables is.

**Definition 5 .**

(equivalence relation ∼). For all ${\overset{⟶}{b}}_{1},{\overset{⟶}{b}}_{2}\in {𝔹}_{k}$, ${\overset{⟶}{b}}_{1}∼{\overset{⟶}{b}}_{2}$ iff $\left\|{\overset{⟶}{b}}_{1}\right\|=\left\|{\overset{⟶}{b}}_{2}\right\|$.

Let ${𝔹}_{k}^{\#}=\left\{\left\|\overset{⟶}{b}\right\|:\overset{⟶}{b}\in {𝔹}_{k}\right\}$. One observes that ∼ partitions *𝔹*_*k*_. If *p* ∈ *𝔹*_*k*_^#^, we use [*p*] to denote the equivalence class whose elements' norms are all *p*.

### 2.3. Probability Distribution

Suppose *𝔹*_*k*_={0,1}^*k*^ is the sampling population. Define a statistic BN on *𝔹*_*k*_ by its binary norm. The range for BN is *𝔹*_*k*_^#^. Define a counting *ρ* : *𝔹*_*k*_^#^⟶*ℕ* by $\rho \left(x\right)=\left|\left\{\overset{⟶}{b}\in {𝔹}_{k}:\left\|\overset{⟶}{b}\right\|=x\right\}\right|$. Now, we could define the probability distribution for BN by prob : *𝔹*_*k*_^#^⟶[0,1] by

(1) $$\begin{array}{c} \text{prob}\left(u\right)=\frac{\rho \left(u\right)}{\sum_{h\in \text{Ran}}\rho \left(h\right)}. \end{array}$$

One observes that

(2) $$\begin{array}{c} \text{prob}\left(u\right)=\frac{\left|\left[u\right]\right|}{\sum_{h\in \text{Ran}}\left|\left[h\right]\right|}. \end{array}$$

This probability distribution reveals the relation between the independent variables and the dependent variables. This would serve our theoretical distribution for our statistical testing *H*_0_: the economic freedom and the death of COVID-19 has no significant relation, i.e., the economic freedom has no great impact on the death of COVID-19. For a concrete construction of such probability distribution, one could refer to Section 6.1.

### 2.4. Metric

A metric or a distance function is a non-negative function *d* on *X* × *X* satisfying identity, symmetry, and triangle properties. In this article, it suffices to define a metric on a closed interval of real number. Fix *I*=[*a*, *b*]⊆*ℝ*, where *a*, *b* ∈ *ℝ* and *a* < *b*. Let $\overset{⟶}{v}$ be a finite vector whose first element is *a*, last element is *b*, and all the other elements are incrementally increased and lie between *a* and *b*. Let FIN[*a*, *b*] be the set of all such vectors. Let $\overset{⟶}{v}=\left(a,v_{2},\ldots ,v_{m-1},b\right),\overset{⟶}{w}=\left(a,w_{2},w_{3},\ldots ,w_{n-1},b\right)\in \text{Fin}\left[a,b\right]$ be arbitrary. Let $\overset{⟶}{v}⊓\overset{⟶}{w}$ denote the vector *q*=(*a*, *q*_1_, *q*_2_,…, *q*_*h*−1_, *b*) whose elements are the projections from $\overset{⟶}{v}$ and $\overset{⟶}{w}$. One observes that FIN[*a*, *b*] is closed under ⊓.

**Definition 6 .**

(atomic norm)${\left\|\overset{⟶}{v}\right\|}_{E}=$

(3) $$\begin{array}{c} \sqrt{{\left(v_{2}-a\right)}^{2}+{\left(v_{3}-v_{2}\right)}^{2}+{\left(v_{4}-v_{3}\right)}^{2}+\cdots {\left(v_{m-2}-v_{m-1}\right)}^{2}+{\left(b-v_{m-1}\right)}^{2}}. \end{array}$$

**Definition 7 .**

(metric). Define *d* : FIN[*a*, *b*] × FIN[*a*, *b*]⟶*ℝ*^+^ by

(4) $$\begin{array}{c} d\left(\overset{⟶}{v},\overset{⟶}{w}\right)=\frac{{\left\|\overset{⟶}{v}\right\|}_{E}+{\left\|\overset{⟶}{w}\right\|}_{E}}{2}-{\left\|\overset{⟶}{v}⊓\overset{⟶}{w}\right\|}_{E}. \end{array}$$

**Example 5 .**

Suppose the closed interval *I*=[0,20] and $\overset{⟶}{v}=\left(0,2,4,8,19,20\right)$ and $\overset{⟶}{w}=\left(0,1,4,6,12,14,15,20\right)$. Then, $\overset{⟶}{v}⊓\overset{⟶}{w}=\left(0,1,2,4,6,8,12,14,15,19,20\right)$. Hence, the norm ${\left\|\overset{⟶}{v}\right\|}_{E}=\sqrt{2^{2}+2^{2}+4^{2}+11^{2}+1^{2}}=\sqrt{146}$; the norm $\overset{⟶}{w}=\sqrt{1^{2}+3^{2}+2^{2}+6^{2}+2^{2}+1^{2}+5^{2}}=\sqrt{80}$; and ${\left\|\overset{⟶}{v}⊓\overset{⟶}{w}\right\|}_{E}=\sqrt{52}$. Thus, $d\left(\overset{⟶}{v}|,|\overset{⟶}{w}\right)=\sqrt{146}+\sqrt{80}/2-\sqrt{52}=3.30$.

**Claim 2 .**

*d* is a metric on FIN[*a*, *b*].

**Proof**

This can be shown by the definitions and some techniques.

This metric will be used in Section 3.3. This metric basically measures the differences between the structures of the attributes in the scoring system. The more similar the structures are, the lower the distances are. Unlike the static Euclidean distance, this metric takes the interval structures into consideration.

### 2.5. Procedures

Let us summarise the whole procedure of our modelling for the sake of data analysis. Let $\overset{⟶}{e}=\left(100,100,100,100,\ldots ,100,100\right)$. Let Death(*C*_*i*_) denote the death rate (or tolls, depending on the context) for the country *i*.

1. Define a metric *d* on a real interval, in particular the transformed interval, an interval for attribute values which lie between 0 and 100, *I*=[0,1200]⊆*ℝ* for the range of attribute values of economic freedom, and calculate $\left\{d\left(\hat{I},{\overset{⟶}{C}}_{i}\right):1\leq i\leq m\right\}$ (one could refer to Section 3.3).
2. Rank *ℂ* via the sorted distances with a rank function *γ*_100_ : *ℂ*⟶{1,2,…, *m*} in which *γ*_*I*_(*C*_*i*_) ≥ *γ*_*I*_(*C*_*j*_) iff $d\left(\overset{⟶}{I},{\overset{⟶}{C}}_{i}\right)\geq d\left(\overset{⟶}{I},{\overset{⟶}{C}}_{i}\right)$.
3. Rank *ℂ* via the sorted distance with a rank function *γ*_88_ in which *γ*_88_(*C*_*i*_) ≥ *γ*_88_(*C*_*j*_) iff Death(*C*_*i*_) ≥ Death(*C*_*j*_).
4. Form the vector $\overset{⟶}{v}={\left(\gamma_{100}{}^{\circ}\gamma_{88}^{-1}\left(l\right)\right)}_{l=1}^{m}$.
5. Convert $\overset{⟶}{v}$ into a sign vector $\text{sg}\left(\overset{⟶}{v}\right):=\left(\chi \left(\overset{⟶}{v}\left(2\right)-\overset{⟶}{v}\left(1\right)\right),\chi \left(\overset{⟶}{v}\left(3\right)-\overset{⟶}{v}\left(2\right)\right),\ldots ,\chi \left(\overset{⟶}{v}\left(m\right)-\overset{⟶}{v}\left(m-1\right)\right)\right)$, where *χ*(*a*)=1 if *a* > 0 and *χ*(*a*)=0 if *a* < 0.
6. Construct the probability distribution for the quotient space *𝔹*_*k*_/∼.
7. Perform statistical testing by locating the position of $\overset{⟶}{v}$ and significant level for the batch of country.
8. Apply the Monte Carlo approach on the sampled batches of countries repeatedly.
9. With the threshold probability 0.5, based on binary distribution for the whole spectrum of statistical testing, perform the overall statistical testing.
10. Draw a conclusion for the relation between *γ*_100_ and *γ*_88_.

## 3. Data Analysis

Following the procedures in Section 2.5, we start to collect, analyse, and produce a report via data analysis. Since the data are huge and hard to handle by the one-off approach, we resort to the sampling technique and reach a conclusion via statistical testing.

### 3.1. Sampling

The raw data consist of 164 countries (we use 1 to 164 to name the countries) up to 2020, June 27^th^. Since the size is too huge, we apply the Monte Carlo approach to sample the 164 countries. We do 20 times (or 20 batches: S1 to S20) sampling with 25 countries over the 164 countries per sampling. The sampled batches are listed in Tables 2 and 3.

### 3.2. Sampled Data

#### 3.2.1. Economic Freedom

Corresponding to the form listed in Table 1, we associate *ℂ* with S1 and define *A*_*ef*_={*A*1, *A*2,…, *A*12}, where *A*1≡Property Rights, *A*2≡Judicial Effectiveness, *A*3≡Government Integrity, *A*4≡Tax Burden, *A*5≡Government Spending, *A*6≡Fiscal Health, *A*7≡Business Freedom, *A*8≡Labor Freedom, *A*9≡Monetary Freedom, *A*10≡Trade Freedom, *A*11≡Investment Freedom, and *A*12≡Financial Freedom. The attribute values are based on a 100-point scoring system [6]. Due to the limitation of space, we list only the first sampling (or S1) regarding its attributes of economic freedom in Table 4. We omit the other 19 similar tables of this form. *A*_ef_ serves as the set of our independent variables.

#### 3.2.2. COVID-19

Now we start to introduce the dependent variables. Indeed we tackle an individual dependent variable each time. Since the data are huge, we only extract the data [7] for sampling one (or S1) as shown in Table 5. Corresponding to the form listed in Table 1, we associate *ℂ* with S1 and define *B*_1_≡ Total Confirmed COVID-19 Cases, *B*_2_≡ Death Toll of COVID-19, *B*_3_≡ Total Recovered COVID-19 Cases, and *B*_4_≡ Population of the Countries. Due to the limitation of space, we list only the first sampling (or S1) regarding its dependent variables. We omit the other 19 similar tables of this form. Moreover, in the later analysis, we only take and fix *B*_2_ as our dependent variable. If the readers are interested in other dependent variables (or *B*_1_, *B*_3_, or other mixed forms), they could simply follow the same approach provided in this article.

### 3.3. Metric

Since we have defined an interval metric in Section 2.4, we could apply it over here. Here we measure the distance between every sampled data and the fixed reference vector $\overset{⟶}{e}=\left(100,200,\ldots ,1100,1200\right)$. We construct the distances for the 164 countries based on economic freedom (for example, the data of sample one could be referred from Table 4) in Tables 6 and 7. Since all the data are presented in the form of 100-point score for the attribute values in Table 4, we need to transform the values in the table to the interval *I*=[0,1200]. For example, the reference vector $\overset{⟶}{e}$ (we still use $\overset{⟶}{e}$ to represent to newly transformed vector) will be $\overset{⟶}{e}=\left(0,100,200,300,\ldots ,1100,1200\right)$. Each country *C* sampled in S1 will be transformed into $\overset{⟶}{C}$, for example, ${\overset{⟶}{\underline{C}}}_{11}\equiv \overset{⟶}{68}=\left(0,64.8,145.7,247.5,379.9,\ldots ,1170,1200\right)$ are the converted data for the first country sampled in the first sampling or country 68. The economic freedom vector for each sampled country is converted by the same way. The converted data are not tabulated. Then, we apply *d* in Section 2.4 on the converted data and repeat the whole processes for other samplings. The complete results regarding the distance for the 20 sampled countries are presented in Tables 6 and 7. The (*i*, *j*) cell in the tables means the value $d\left(\overset{⟶}{e},{\overset{⟶}{\underline{C}}}_{ij}\right)$, where ${\underline{C}}_{ij}$ denotes the *i*-th country sampled in *j*-th sampling and ${\overset{⟶}{\underline{C}}}_{ij}$ denotes the converted data for ${\underline{C}}_{ij}$.

## 4. Absolute Reference

By the derived distances presented in Tables 6 and 7, we could construct absolute references. The absolute references would server as the benchmarks for other internal structures. Let us use *ℂ*_*s*_ to denote the set of sampled countries in *s*-th sampling. Let ${\overset{⟶}{\underline{C}}}_{si},{\overset{⟶}{\underline{C}}}_{sj}\in {\mathbb{C}}_{s}$ be arbitrary.

**Definition 8 .**

(ordering of the sampled countries). ${\underline{C}}_{is}\geq {\underline{C}}_{js}$ iff $d\left(\overset{⟶}{e},{\overset{⟶}{\underline{C}}}_{is}\right)\geq d\left(\overset{⟶}{e},{\overset{⟶}{\underline{C}}}_{js}\right)$.

Based on this ordering, we could generate the absolute references (Tables 8 and 9). Let us take S1 for example: *C*_68_ > *C*_112_ > *C*_92_ > ⋯>*C*_41_ > *C*_85_ > *C*_14_. From these absolute references (or ordering for the samplings), we could view the structure (or interval) difference between the ideal scoring (or $\overset{⟶}{e}$) and real scoring results. Indeed, an absolute reference is a reference acting like ordering without specific scales. Such reference is useful when the precise values are unknown or when the precision of the data is questionable. In this article, we use relative distances between a country's economic freedom and others to create such ordering.

## 5. Ordering for COVID-19 Fatalities

Based on Table 5 and other omitted tables, we start to construct the ordering (or ranking) based on the fatalities of COVID-19.

**Definition 9 .**

(ordering on fatalities). ${\underline{C}}_{is}\geq {\underline{C}}_{js}$ iff $\text{Death}\left({\underline{C}}_{is}\right)\geq \text{Death}\left({\underline{C}}_{js}\right)$, where $\text{Death}\left({\underline{C}}_{is}\right)$ is the death toll for *i*-th country sampled in *s*-th sampling.

Based on this ordering, we have the results presented in Tables 10 and 11. Let us take the cells in S1 for example: *C*_78_ > *C*_98_ > *C*_76_ > ⋯>*C*_14_ > *C*_99_ > *C*_21_.

## 6. Norm and Probability

In this experiment, we only consider *N*=23 and construct its distribution accordingly. Hence, the domain is {0,1}^23^ and the range lies between 0 and 2^23^ − 1=8388607 (indeed some of the values' probability is 0). This section generalises Example 3. The higher the value is, the higher the impact of independent variables on dependent variable is.

### 6.1. Probability Distribution

We have already constructed the theoretical setting of probability distribution for our testing in Section 2.3. Based on that framework and the data given, we could create the theoretical probability distribution prob in Figure 1.

The (one-tailed) critical values for 5 and 10 percentages are 138 and 78 (via numerical computation), respectively; that is, if the sampled value is larger than the critical values, we should reject *H*_*o*_: there is no significant relation between the economic freedom and death of COVID-19.

### 6.2. Real Results

In comparison with the absolute reference, we could generate the binary sign vectors for the real data from each sampling *S*_*j*_ (or simply *j*) in Table 12—for the formula and explanation of sign vectors, one could refer to Section 2.2. However, in these 0 and 1 representations, it separates the proportional and inversely proportional relation between the economic freedom and death of COVID-19. To take all the factors into consideration, one further analyses the alternative behaviour of 0 and 1. If there are too many alternations between 0 and 1, it would indicate that there is a less relation between those two. On the other hand, if the alternative times are few, then it leads to the longer length of subvector consisting of pure 1. The alternative results are shown in Table 13.

Based on Table 13 and definitions in Section 2.2, we could compute the binary norm for each sampling batch *S*_*j*_ (or *J*) as shown in Table 14.

## 7. Conclusion and Future Work

The contribution of death in COVID-19 is very complicated. We use economic freedom to capture a potential factor in such contribution. To verify the truth of great impact from economic freedom, we devise a metric, two norms, absolute ordering, binary ordering, and probability distribution for the statistical testing population. Based on our research, we find out that the economic freedom has no significant relation to the death of COVID-19. This might provide some reference for the decision makers of the countries. In the future research, one could further study the relation between economic freedom and other ratios related to COVID-19. One could also use other nonparametric approaches to enrich the statistical testing. There is another related paper on the same topic [8]. In that paper, the authors use two-step estimators: negative binomial regression and nonlinear least squares, and find out there is a close relation between economic freedom and fatalities of COVID-19. In essence, their approach focuses more on statistical techniques, while ours focuses more on mathematical approaches. For the future researcher, he could compare or combine these methods to yield a comprehensive or generalised theory that could accommodate and single out the factors that cause the discrepancies.

## Figures and Tables

**Figure 1:** Theoretical distribution of binary norm.

**Table 1:** Independent-dependent analysis.

Countries	*A*_1_	*A*_2_	…	*A*_*p*_	*B*_1_	*B*_2_	…	*B*_*q*_
*C*_1_	*a*_11_	*a*_12_	…	*a*_1*p*_	*b*_11_	*b*_12_	…	*B*_1*q*_
*C*_2_	*a*_21_	*a*_22_	…	*a*_2*p*_	*b*_21_	*b*_22_	…	*b*_2*q*_
…								
*C*_*m*_	*a*_*m*1_	*a*_*m*2_	…	*a*_*mp*_	*b*_*m*1_	*b*_*m*2_	…	*b*_*mq*_

**Table 2:** 20 sampled batches—S1 to S10.

Order	S1	S2	S3	S4	S5	S6	S7	S8	S9	S10
1	68	25	69	10	27	65	72	56	64	163
2	141	127	93	98	55	85	75	151	150	19
3	21	95	5	56	14	115	159	112	65	10
4	129	41	30	45	7	35	130	136	9	117
5	127	17	151	74	119	57	128	139	69	52
6	99	151	33	89	20	160	147	100	27	18
7	89	14	156	26	124	95	19	27	113	88
8	2	43	132	73	35	118	122	83	53	65
9	128	76	44	84	153	29	129	16	84	105
10	108	28	48	70	150	15	9	47	110	150
11	112	62	126	67	151	71	118	134	156	26
12	92	131	6	121	90	86	91	87	89	161
13	98	10	46	69	80	89	39	107	52	82
14	18	119	84	50	37	50	71	52	21	27
15	148	128	39	97	84	13	81	111	132	57
16	124	121	34	3	45	56	15	48	15	29
17	1	18	95	92	75	91	158	101	66	20
18	32	16	98	18	113	41	125	46	127	116
19	76	92	26	87	59	7	144	113	56	38
20	14	42	85	142	85	32	46	70	97	41
21	41	60	1	37	48	61	21	76	140	92
22	137	103	144	137	38	75	86	84	102	128
23	85	120	53	2	132	124	132	119	31	7
24	78	163	117	122	111	122	99	74	163	22
25	52	118	62	77	66	19	35	123	88	103

**Table 3:** 20 sampled batches—S11 to S20.

Order	S11	S12	S13	S14	S15	S16	S17	S18	S19	S20
1	76	91	83	59	64	119	129	154	15	37
2	23	124	53	63	46	123	8	82	30	55
3	29	151	126	24	143	137	6	35	43	119
4	12	126	129	55	53	108	122	4	148	163
5	73	65	9	143	86	54	152	40	76	155
6	157	86	18	100	59	76	7	69	133	18
7	49	54	102	50	40	6	120	19	8	6
8	68	119	50	85	52	156	93	89	146	99
9	15	87	104	74	32	152	70	146	145	122
10	48	8	74	40	68	111	27	143	57	162
11	104	11	87	115	36	101	25	134	26	25
12	99	67	125	79	135	85	136	70	101	156
13	142	59	158	52	156	3	66	38	131	147
14	136	139	20	159	39	37	110	61	31	10
15	41	43	57	69	96	30	67	20	20	134
16	115	148	151	108	50	66	50	142	6	79
17	151	56	54	49	27	51	53	54	63	44
18	77	15	27	36	47	162	26	98	25	157
19	126	16	90	136	154	124	132	56	70	4
20	108	82	93	87	132	95	89	151	85	20
21	95	39	161	98	138	138	44	111	71	67
22	60	37	44	21	62	120	76	113	118	153
23	36	6	16	54	120	69	141	108	84	97
24	1	42	86	109	12	134	84	7	41	148
25	74	10	103	119	157	136	73	52	58	136

**Table 4:** Sample one for economic freedom.

S1	*A*1	*A*2	*A*3	*A*4	*A*5	*A*6	*A*7	*A*8	*A*9	*A*10	*A*11	*A*12
68	64.8	45.7	47.5	79.9	34.5	83.6	60.2	64.6	79.9	86.4	80	70
141	33.7	20.8	25.5	86.1	94.5	12.4	53.5	60	77	52	5	20
21	57.3	46.7	45.6	70.4	54.6	4.6	60.5	49.5	77.2	67.8	60	50
129	64.6	72.3	49.6	99.8	61.8	19.3	66.6	63.3	81	75.4	45	50
127	69.8	62.6	41.8	76.9	80.6	83.8	76.7	66.4	82	73.2	65	40
99	58.3	34.7	36.7	76.1	79.3	87.5	67	58.4	70.9	87.6	75	60
89	86.4	74.4	90.3	64.1	45.4	99	66.8	45.3	76.4	86.4	95	80
2	57.1	33	38.8	85.9	74.6	86.3	65.7	52.1	81.2	88.4	70	70
128	41	26.5	37.4	88.3	77.1	73	64.8	43.4	68.1	64.2	60	30
108	93.3	79.1	93.9	71	57.8	98.3	90.4	86.7	87	92.2	80	80
112	62.5	42.7	42.2	91.5	71	87.7	80.6	67	77.7	86.2	65	60
92	43.1	42.1	24.8	79	71.7	23.6	41.9	62.8	69.1	75.4	50	50
8	75.8	62.6	53.3	91.5	82.1	79.3	82.5	60.2	73.8	88.2	80	70
18	20.1	11.2	23.1	86.3	54.2	14.2	58.3	52.9	69.9	67.8	15	40
148	59.5	48	43.4	80.7	85.9	96.4	83	63.7	74	83	55	60
124	72.5	56.1	55.1	90.3	70.4	85.6	58.6	63	78.1	86.4	70	50
1	48.3	30	24.8	91.4	79.2	99.9	54.7	61.6	81	66	10	10
32	69.9	61.1	73.4	76.4	80.8	90.5	75	64.7	85.2	89	85	70
76	62.1	50.5	46.8	80	74.8	80.2	77.7	74	77.7	68.4	80	50
14	84.5	62.5	80.2	46.7	17.2	77	75.2	61.1	80.5	86.4	85	70
41	86.3	84.6	93	42	19.7	97.7	88.7	86.2	84.6	86.4	90	80
137	58.4	38	46.6	63.7	67.4	64	62	58.8	75.9	75.8	45	50
85	44.6	30.8	25	90.8	72.5	0	45.6	47.8	75.6	77.4	60	50
78	64.8	54.6	49.6	91.8	73.5	55.9	60.1	52.5	77.6	81.2	70	60
52	36.5	45.1	29.4	77.4	90.8	79.2	48.6	57.6	62.7	60.8	35	20

**Table 5:** Sample one for COVID-19.

S1	*ℂ*	*B*_1_	*B*_2_	*B*_3_	*B*_4_
68	Hungary	4127	578	2663	9660521
141	Sudan	9257	572	4014	43828543
21	Brazil	1280054	56109	697526	212541690
129	Senegal	6354	98	4193	16734279
127	Sao Tome and Principe	712	13	219	219087
99	Mexico	208392	25779	120562	128914507
89	Luxembourg	4173	110	3968	625810
2	Albania	2269	51	1298	2877821
128	Saudi Arabia	174577	1474	120471	34805142
108	New Zealand	1520	22	1484	5002100
112	North Macedonia	5758	268	2206	2083375
92	Malawi	1005	13	260	19119281
98	Mauritius	341	10	326	1271749
18	Bolivia	28503	913	7338	11670618
148	Thailand	3162	58	3040	69798329
124	Romania	25697	1579	18181	19238321
1	Afghanistan	30451	683	10306	38910996
32	Chile	263360	5068	223431	19114153
76	Jamaica	686	10	539	2961033
14	Belgium	61106	9731	16918	11589102
41	Denmark	12675	604	11508	5792000
137	South Africa	124590	2340	64111	59297807
85	Lebanon	1697	33	1144	6825627
78	Jordan	1104	9	830	10201800
52	Ethiopia	5425	89	1688	114903773

**Table 6:** Distance function for 20 samplings—S1 to S10.

S1	S2	S3	S4	S5	S6	S7	S8	S9	S10
61.0	80.1	82.2	74.2	78.3	73.2	53.9	59.2	66.8	72.2
76.2	76.8	75.4	72.4	73.6	84.0	72.8	83.4	80.4	71.3
70.7	72.4	71.1	59.2	85.1	68.6	66.5	62.3	73.2	74.2
80.8	82.1	71.4	82.3	64.9	77.2	74.3	85.7	70.2	65.0
76.8	71.8	83.4	78.5	72.8	67.1	76.9	78.9	82.2	80.7
75.0	83.4	69.7	65.5	84.4	49.2	67.7	77.4	78.3	75.8
65.5	85.1	57.3	71.3	71.1	72.4	71.3	78.3	74.4	61.8
80.4	70.4	74.8	68.7	77.2	65.0	67.8	67.3	57.5	73.2
76.9	69.5	81.5	74.8	73.1	71.8	80.8	73.1	74.8	68.1
73.3	61.3	60.1	71.4	80.4	83.2	70.2	72.3	72.7	80.4
62.3	73.8	71.9	76.5	83.4	64.2	65.0	77.6	57.3	71.3
63.0	74.9	49.9	77.8	71.9	80.1	82.6	62.7	65.5	82.3
72.4	74.2	74.0	82.2	78.4	65.5	66.0	45.7	80.7	72.5
75.8	72.8	74.8	79.9	54.1	79.9	64.2	80.7	70.7	78.3
68.8	76.9	66.0	65.1	74.8	70.4	74.4	69.2	74.8	67.1
71.1	77.8	77.3	71.4	82.3	59.2	83.2	60.1	83.2	71.8
71.3	75.8	72.4	63.0	72.8	82.6	71.6	75.4	33.6	84.4
74.3	73.1	72.4	75.8	74.4	82.1	68.8	74.0	76.8	74.5
69.5	63.0	71.3	62.7	82.6	64.9	59.4	74.4	59.2	74.0
85.1	77.7	84.0	59.7	84.0	74.3	74.0	71.4	65.1	82.1
82.1	66.0	71.3	54.1	60.1	72.0	70.7	69.5	64.2	63.0
67.7	82.7	59.4	67.7	74.0	72.8	80.1	74.8	82.3	76.9
84.0	73.3	57.5	80.4	74.8	71.1	74.8	72.8	60.9	64.9
67.7	72.2	65.0	67.8	69.2	67.8	75.0	78.5	72.2	68.2
80.7	65.0	73.8	78.6	33.6	71.3	77.2	72.3	61.8	82.7

**Table 7:** Distance function for 20 samplings—S11 to S20.

S11	S12	S13	S14	S15	S16	S17	S18	S19	S20
69.5	82.6	67.3	82.6	66.8	72.8	80.8	81.1	83.2	54.1
82.3	71.1	57.5	83.2	74.0	72.3	71.6	72.5	71.4	73.6
71.8	83.4	71.9	74.4	52.9	67.7	49.9	77.2	70.4	72.8
68.7	71.9	80.8	73.6	57.5	73.3	67.8	90.3	68.8	72.2
68.7	73.2	70.2	52.9	80.1	71.6	80.6	49.1	69.5	58.9
62.9	80.1	75.8	77.4	82.6	69.5	64.9	82.2	32.3	75.8
59.6	71.6	82.3	79.9	49.1	49.9	73.3	71.3	71.6	49.9
61.0	72.8	79.9	84.0	80.7	57.3	75.4	65.5	73.5	75.0
83.2	62.7	78.8	78.5	74.3	80.6	71.4	73.5	80.1	67.8
60.1	71.6	78.5	49.1	61.0	69.2	78.3	52.9	67.1	82.0
78.8	84.0	62.7	68.6	80.7	75.4	80.1	77.6	71.3	80.1
75.0	76.5	68.8	83.9	74.5	84.0	85.7	71.4	75.4	57.3
59.7	82.6	71.6	80.7	57.3	71.4	33.6	74.0	74.9	67.7
85.7	78.9	84.4	66.5	66.0	54.1	72.7	72.0	60.9	74.2
82.1	70.4	67.1	82.2	72.7	71.4	76.5	84.4	84.4	77.6
68.6	68.8	83.4	73.3	79.9	33.6	79.9	59.7	49.9	83.9
83.4	59.2	71.6	59.6	78.3	74.1	57.5	71.6	83.2	81.5
78.6	83.2	78.3	80.7	72.3	82.0	71.3	72.4	80.1	62.9
71.9	73.1	71.9	85.7	81.1	71.1	74.8	59.2	71.4	90.3
73.3	72.5	75.4	62.7	74.8	72.4	65.5	83.4	84.0	84.4
72.4	66.0	82.3	72.4	78.2	78.2	81.5	69.2	64.2	76.5
66.0	54.1	81.5	70.7	73.8	73.3	69.5	74.4	65.0	73.1
80.7	49.9	73.1	71.6	73.3	82.2	76.2	73.3	74.8	65.1
71.3	77.7	80.1	84.7	68.7	77.6	74.8	64.9	82.1	68.8
78.5	74.2	82.7	72.8	62.9	85.7	68.7	80.7	82.9	85.7

**Table 8:** Absolute references for 20 samplings—S1 to S10.

S1	S2	S3	S4	S5	S6	S7	S8	S9	S10
68	28	6	37	66	160	72	107	66	88
112	92	156	56	37	56	144	56	156	92
92	118	53	142	48	71	71	48	53	7
89	60	144	87	7	7	118	112	56	117
78	76	48	92	111	118	39	87	31	57
137	43	117	97	124	89	159	83	88	105
148	17	39	89	90	57	147	111	140	22
76	163	33	137	75	122	122	76	97	26
21	95	5	122	119	115	125	70	89	19
124	119	1	73	153	13	9	123	64	29
1	16	26	26	55	124	21	47	9	163
98	120	30	70	38	19	19	119	21	82
108	62	126	3	113	29	158	16	163	65
32	10	98	98	132	61	75	46	110	38
99	131	95	10	84	95	46	113	65	10
18	18	62	84	35	75	130	84	113	116
141	127	46	18	27	65	81	101	132	18
127	128	132	67	80	32	132	100	84	128
128	42	84	121	150	35	99	134	127	27
2	121	93	74	45	50	128	27	27	150
52	25	34	77	59	86	35	74	150	52
129	41	44	50	151	41	86	139	52	41
41	103	69	2	85	91	129	52	69	161
85	151	151	69	20	15	91	151	102	103
14	14	85	45	14	85	15	136	15	20

**Table 9:** Absolute references for 20 samplings—S11 to S20.

S11	S12	S13	S14	S15	S16	S17	S18	S19	S20
49	6	53	40	40	66	66	40	133	6
142	37	87	143	143	6	6	143	6	37
48	56	57	49	156	37	53	56	31	156
68	87	83	87	53	156	7	142	71	155
157	39	125	159	68	137	89	7	118	157
60	148	9	115	157	111	122	89	57	97
115	43	158	21	39	76	73	111	148	147
73	124	54	54	64	124	76	19	76	122
12	8	126	98	12	30	26	70	43	148
76	54	90	119	47	3	70	54	26	163
1	126	16	108	96	54	8	61	70	119
29	82	93	55	120	123	110	98	30	153
126	119	18	24	62	95	120	82	8	55
95	16	27	100	46	119	132	108	146	10
108	65	74	74	32	120	84	146	84	99
99	10	104	50	135	108	93	38	131	18
74	67	50	52	132	51	141	113	101	67
77	42	86	36	138	101	67	35	145	134
104	139	129	69	27	134	27	134	25	25
36	86	44	59	50	138	50	52	41	44
41	91	102	63	86	152	25	154	58	162
23	59	161	79	52	162	152	69	63	79
15	15	103	85	36	69	129	151	15	20
151	151	151	109	154	85	44	20	85	136
136	11	20	136	59	136	136	4	20	4

**Table 10:** Ordering for each batch based on death toll of COVID-19—S1 to S10.

S1	S2	S3	S4	S5	S6	S7	S8	S9	S10
78	43	53	67	90	15	15	83	53	117
98	131	117	98	20	35	35	101	15	20
76	25	126	26	35	118	118	151	102	22
127	151	151	69	151	57	91	76	69	26
92	17	69	142	150	91	39	16	140	92
108	76	98	92	84	160	147	134	64	150
85	127	26	84	48	85	159	84	127	57
2	92	39	87	85	56	132	48	150	163
148	118	62	56	132	50	129	87	163	161
52	16	84	2	38	65	19	56	84	82
129	163	48	50	59	7	9	52	56	10
89	62	85	10	7	89	130	136	132	88
112	42	30	37	37	95	81	123	110	38
141	10	132	89	80	19	128	47	31	52
68	95	95	97	113	13	122	113	88	65
41	60	93	74	66	41	144	112	52	7
1	103	156	3	111	61	46	74	65	19
18	28	6	18	124	122	71	100	89	103
128	41	1	77	45	124	125	111	97	116
124	18	44	121	153	71	72	46	9	41
137	120	5	122	119	115	99	107	113	18
32	121	144	73	14	32	75	119	156	128
14	128	46	137	55	29	21	70	66	29
99	119	34	45	75	75	158	139	21	105
21	14	33	70	27	86	86	27	27	27

**Table 11:** Ordering for each batch based on death toll of COVID-19—S11 to S20.

S11	S12	S13	S14	S15	S16	S17	S18	S19	S20
49	43	83	49	53	101	53	20	43	162
15	126	53	69	12	162	25	35	101	25
126	15	90	98	96	51	67	151	131	20
104	67	20	36	64	76	26	4	20	67
12	151	126	63	36	69	76	69	25	4
151	16	104	108	39	134	84	142	15	134
76	91	151	159	135	108	152	98	145	163
142	39	102	85	62	85	132	134	76	147
36	87	57	87	132	30	110	108	26	148
108	56	16	24	50	152	50	56	118	10
48	82	87	50	52	37	129	82	57	37
136	42	161	109	59	123	7	146	63	136
95	148	50	52	47	136	136	38	133	97
60	10	129	59	138	95	89	52	84	79
23	65	93	136	156	138	93	7	85	156
74	59	9	79	40	156	6	89	30	6
68	37	103	74	68	54	66	19	146	44
41	54	74	54	120	6	141	113	148	18
1	6	54	40	46	66	8	54	31	155
77	8	44	100	32	111	44	40	6	122
73	124	18	115	143	3	120	111	41	153
115	11	125	143	157	120	122	61	8	119
29	119	158	119	86	124	73	143	71	99
99	139	27	55	27	137	70	70	58	55
157	86	86	21	154	119	27	154	70	157

**Table 12:** Sign vectors.

1	2	3	4	5	6	7	8	9	10	11	12	13	14	15	16	17	18	19	20
1	1	1	0	1	0	0	1	1	1	1	1	0	1	1	1	1	0	1	0
0	1	1	0	0	0	0	1	0	0	0	1	1	0	1	0	0	1	0	1
1	1	1	1	1	1	1	0	0	1	1	0	1	1	0	0	0	1	1	0
0	0	0	0	0	1	0	1	0	0	0	1	0	1	1	1	0	0	0	1
1	0	0	1	0	0	1	1	1	1	1	0	1	0	0	0	1	0	1	0
1	1	0	1	0	1	0	0	1	0	0	1	1	0	1	0	1	1	0	0
0	0	0	0	1	0	1	0	1	1	0	0	0	1	0	1	0	1	0	0
0	1	1	0	0	1	1	1	0	1	1	0	0	0	1	0	0	0	1	1
1	1	1	1	0	0	0	0	1	0	0	0	1	1	1	1	1	0	0	1
1	0	0	0	1	0	0	1	0	1	0	1	0	1	1	0	1	1	1	0
0	1	1	0	0	1	1	1	1	0	1	1	1	1	1	1	0	1	1	1
0	1	0	0	0	1	1	0	0	1	0	0	0	0	0	1	1	1	0	0
1	0	1	1	1	0	1	1	0	1	0	1	1	1	1	0	0	1	1	1
0	0	0	0	0	0	0	1	1	0	1	0	0	1	0	1	1	0	1	0
1	0	1	1	0	1	0	0	1	0	0	1	0	0	0	0	0	1	0	0
0	1	0	0	1	0	1	1	0	1	0	0	1	0	1	1	0	1	1	1
1	0	0	1	1	0	0	0	0	1	1	1	0	0	1	0	1	1	0	0
1	1	1	1	1	1	1	0	0	0	0	0	0	0	1	0	0	0	0	0
0	0	1	0	0	0	0	1	1	1	1	1	1	1	1	1	1	0	0	1
0	0	0	0	0	1	1	0	1	0	0	0	0	0	0	1	0	1	1	1
1	1	0	1	1	1	0	1	0	1	0	1	0	0	1	1	0	1	0	0
1	0	1	0	0	0	0	0	0	0	1	0	1	1	1	0	1	0	0	1
0	0	1	1	0	1	1	1	1	0	1	1	1	1	0	0	1	1	1	0
0	1	0	0	1	1	1	0	1	1	0	1	1	0	1	1	1	1	0	0

**Table 13:** Relational vectors.

1	2	3	4	5	6	7	8	9	10	11	12	13	14	15	16	17	18	19	20
0	1	1	1	0	1	1	1	0	0	0	1	0	0	1	0	0	0	0	0
0	1	1	0	0	0	0	0	1	0	0	0	1	0	0	1	1	1	0	0
0	0	0	0	0	1	0	0	1	0	0	0	0	1	0	0	1	0	0	0
0	1	1	0	1	0	0	1	0	0	0	0	0	0	0	0	0	1	0	0
1	0	1	1	1	0	0	0	1	0	0	0	1	1	0	1	1	0	0	1
0	0	1	0	0	0	0	1	1	0	1	0	0	0	0	0	0	1	1	1
1	0	0	1	0	0	1	0	0	1	0	1	1	0	0	0	1	0	0	0
0	1	1	0	1	0	0	0	0	0	0	1	0	0	1	0	0	1	0	1
1	0	0	0	0	1	1	0	0	0	1	0	0	1	1	0	1	0	0	0
0	0	0	1	0	0	0	1	0	0	0	1	0	1	1	0	0	1	1	0
1	1	0	1	1	1	1	0	0	0	0	0	0	0	0	1	0	1	0	0
0	0	0	0	0	0	1	0	1	1	1	0	0	0	0	0	0	1	0	0
0	1	0	0	0	1	0	1	0	0	0	0	0	1	0	0	0	0	1	0
0	1	0	0	1	0	1	0	1	1	0	0	1	0	1	0	0	0	0	1
0	0	0	0	0	0	0	0	0	0	1	0	0	1	0	0	1	1	0	0
0	0	1	0	1	1	0	0	1	1	0	0	0	1	1	0	0	1	0	0
1	0	0	1	1	0	0	1	1	0	0	0	1	1	1	1	0	0	1	1
0	0	1	0	0	0	0	0	0	0	0	0	0	0	1	0	0	1	1	0
1	1	0	1	1	0	0	0	1	0	0	0	0	0	0	1	0	0	0	1
0	0	1	0	0	1	0	0	0	0	1	0	1	1	0	1	1	1	0	0
1	0	0	0	0	0	1	0	1	0	0	0	0	0	1	0	0	0	1	0
0	1	1	0	1	0	0	0	0	1	1	0	1	1	0	1	1	0	0	0
1	0	0	0	0	1	1	0	1	0	0	1	1	0	0	0	1	1	0	1

**Table 14:** Binary norm for the 20 samplings: S1 to S20.

1	2	3	4	5	6	7	8	9	10	11	12	13	14	15	16	17	18	19	20
8	11	15	8	11	8	9	6	14	5	6	6	9	15	17	8	11	17	7	8

## Data Availability

The data supporting the findings of this study are included within the article.
